The article "Double Pump Sequential Constant Citrate Anticoagulation in General Hemodialysis" was retracted in 2023. Reasons: signs of a paper mill; compromised peer review; unreliable results or conclusions.

# Double Pump Sequential Constant Citrate Anticoagulation in General Hemodialysis

**DOI:** 10.1155/2022/6047074

**Published:** 2022-07-26

**Authors:** Li Tang, Jiali Zhang, Qijun Cheng, Jie Li, Ling Zhou, Li Wang, Changbin Liao

**Affiliations:** ^1^Zigong Third People's Hospital, Sichuan 643000, China; ^2^Zigong First People's Hospital, Sichuan 643000, China

## Abstract

**Objective:**

To investigate the safety and efficacy of single-pump and double-pump sequential anticoagulation in general hemodialysis under the condition of constant citrate.

**Methods:**

A total of 32 patients with end-stage renal disease complicated with hemorrhage admitted by Zigong Third People's Hospital from December 2019 to December 2020 were collected. Randomly divided into single pump group (*n* = 17) and double pump group (*n* = 15). The coagulation of dialyzer and intravenous pot was compared between the two groups. Then, the changes of serum calcium before treatment, after 2 h treatment, and after the completion of the treatment, and the front of the blood pump and intravenous pot, as well as behind the intravenous pot were observed and recorded in the two groups. Then, single-pool clearance of urea/volume (spKt/V) was compared between the two groups.

**Results:**

There were few differences in dialyzer coagulation between the single pump group and double pump group. However, the single pump group had a significant increase in the number of intravenous pot coagulations than the double pump group. At 2 h for dialysis, the serum calcium level behind the intravenous pot in the double pump group was notably lower than that in the single pump group. And after the completion of dialysis, the serum calcium returned to pretreatment level. The Kt/v in both groups reached the normal standard without statistically significant difference. And there were no adverse reactions in the patients of both groups after dialysis.

**Conclusion:**

For hemodialysis patients with bleeding, dual-pump segmented anticoagulation is superior to single-pump anticoagulation in intravenous pot anticoagulation. Double pump segmented sequential constant citrate anticoagulation can be utilized as a new simple and effective anticoagulation method for clinical hemodialysis.

## 1. Introduction

Currently, hemodialysis is the most important treatment for patients with end-stage renal disease (ESRD) in China [1]. Due to changes in renal excretion and endocrine function, a range of mineral metabolism disorders occur in patients with end-stage renal disease, including metabolism disorders of calcium and phosphorus [2]. Therefore, good diagnosis and treatment for the metabolism of calcium and phosphorus are the important content for chronic disease management in dialysis patients. The quality of hemodialysis has a significant relationship with the treatment of the disease in patients [3]. And successful hemodialysis relies on adequate anticoagulation. Specifically, anticoagulation maintains the flow of blood in the vascular access and dialyzer and prevents hemodialysis-induced thromboembolic disease [4]. Low molecular weight heparin and heparin injection are the most commonly applied anticoagulants at present. However, the applications of the above conventional anticoagulants aggravate the original bleeding in patients with combined bleeding or high-risk bleeding tendency [5]. In the past, heparin-free hemodialysis was usually chosen, while now, coagulation in dialyzer and tubes has a high incidence, short dialysis time, and low dialysis adequacy. Additionally, it is reported that heparin-free hemodialysis may aggravate the consumption of platelets and reduce the number of platelets, which is not conducive to the control of bleeding [6].

As an extracorporeal anticoagulant, citrate has a reliable anticoagulant effect. And the anticoagulation of citrate is limited to the extracorporeal circuit, which has little effect on coagulation of patients in vivo. Therefore, citrate is especially suitable for patients with bleeding or high-risk bleeding tendency, which can reduce bleeding complications and prolong the service life of the filter [7]. By binding to calcium ions in the plasma, sodium citrate forms a calcium citrate complex, declines the concentration of free calcium ions in plasma, and inhibits coagulation pathways in vitro and vivo, thereby achieving the anticoagulant effect [5]. In 1961, Morita et al. [8] introduced regional trisodium citrate (TSC) anticoagulation as extracorporeal anticoagulant therapy in patients with high-risk bleeding. Evenepoel et al. [9] have demonstrated that dialysate containing calcium can be applied for citrate anticoagulation. Since the use of citrate anticoagulation protocol with calcium-containing dialysate does not require additional calcium supplementation and simplifies the specific operation, simplified-regional citrate anticoagulation (S-RCA) has been carried out in many centers in China [10, 11]. In recent years, various dialysis centers have successively proposed a modified regional citrate anticoagulation (RCA) regimen (two-segment RCA) for better application in maintenance hemodialysis (MHD) patients. Clinically, iCa^2+^ concentrations have been found to be particularly high in venous bubble pools, which would be a critical point for single-pump coagulation [12, 13]. Given this consideration, we transferred 2/3 of the TSC from the prefilter to the RCA-1 based postfilter RCA-2, referred to as the double pump in this experiment. Specifically, citrate is continuously pumped in front of the filter, and a small amount of citrate is added to the intravenous pot. And dialysate containing calcium is applied, so the venous line does not require a calcium supplement. All in all, two-segment RCA has achieved great anticoagulation effect. However, S-RCA does not have a standard operating procedure, so periodic testing of ionized calcium is required to adjust citrate dosage. Heparin anticoagulation in hemodialysis is based on body weight to estimate heparin dosage. It has been reported [12] that the ratio of citrate/blood flow is a key factor affecting the anticoagulant effect of RCA in general hemodialysis. We are therefore curious whether effective anticoagulation can be achieved by setting a constant citrate/blood flow ratio. Currently, RCA has been applied as the anticoagulant method for continuous renal replacement therapy for acute kidney injury in the clinical. However, RCA has not been widely carried out in general hemodialysis patients. At present, a few centers in China have carried out RCA, but each center has different dialysate calcium ion concentration and different citrate concentration selection due to the lack of standardized operating guiding in general hemodialysis. Therefore, this study is intended to compare the safety and efficacy of single-pump and double-pump sequential anticoagulation in general hemodialysis by constant fixation of citrate dose.

## 2. Materials and Methods

### 2.1. Study Subjects

A total of 32 patients with ESRD complicated with bleeding or high-risk bleeding admitted by Zigong Third People's Hospital from December 2019 to December 2020 were collected. High risk of bleeding [12] was defined as active bleeding (within 3 days), preinfiltrative surgery (within 7 days) and postoperative (within 3 days). Patients were randomized into single-pump group (*n* = 17) and double-pump group (*n* = 15). The difference was that the double pump group transferred 2/3 of the TSC from the prefilter to the RCA-1 based postfilter RCA-2. The details of the method are shown in Figure 1.

Criteria inclusion of the patients was shown as follows: (1) patients complicated with bleeding or high-risk bleeding and with heparin contraindications; (2) patients who were informed and agreed with the study and signed informed consent. Exclusion criteria were shown as follows: (1) blood pressure was less than 90/60 mmHg; (2) patients with abnormal liver function, and patients whose elevation of transaminase and total bilirubin were two times higher than normal values; (3) oxygen saturation was less than 90%; (4) patients younger than 18 years and older than 95 years; (5) single ultrafiltration volume was higher than 3000 ml. All patients or their clients obtained and signed written informed consent. This study was approved by the Ethics Committee of Zigong Third People's Hospital.

### 2.2. Treatment Methods

The Fresenius 4008 s dialysis machine was applied for 4 h general hemodialysis treatment without vascular access restriction. Polyflux 14 L (Gambro) was carried out as the dialyzer. Dialysate ion concentration was shown as follows: sodium 138 mmol/L, potassium 2 mmol/L, calcium 1.5 mmol/L, magnesium 0.5 mmol/L, chlorine 109.5 mmol/L, and bicarbonate radical 35 mmol/L. The dialysis blood flow was controlled at 200 ml/min, and the citrate dosage was set at 1.3 times the blood flow. After 3 h, the citrate stopped. Then, blood flow was controlled at 250 ml/min after citrate stopped.

Additionally, 4% citrate was pumped at 260 ml/h from a reducing tee in the arterial line in single pump and at 175 ml/h in double pump, and at 85 ml/min from the front of intravenous pot. Citrate dosage was not adjusted during dialysis, and citrate was discontinued if postfilter calcium concentration was below 0.3 mmol/l. Specific treatments were shown in Figure 1. All patients completed 104 general hemodialysis treatments with citrate anticoagulation. Specifically, the single pump group was completed 54 times, and the double pump group was 50 times. Blood gas analysis was recorded before dialysis, 2 h after dialysis and at the completion of dialysis in both groups. As Figure 1 showed, before citrate application, predialysis ① blood gas analysis was collected; at 2 h after dialysis and at the completion of dialysis, ② ③ blood gas analysis (all pumps were open) was first collected, and after stopping citrate pump for 5 min, ① blood gas analysis was collected.

### 2.3. Detection of Dialysis Indicators

The urea concentration and total excretion amount of exudate, as well as the serum urea concentration and distribution volume during dialysis, were recorded in all patients. Then, single-pool clearance of urea/volume (spKt/V) was calculated and compared between the two groups. Additionally, spKt/v≧1.2 was sufficient for dialysis [14].

### 2.4. Coagulation Profile Score

The coagulation of dialyzer and intravenous pot during dialysis was observed and compared between the two groups. The degree of clotting in the dialyzer was scored semiquantitatively with reference to a scoring system [15]. Grade 0, no clotting detected; grade 1, small amount of clot formation (presence of fibrous rings); grade 2, clot formation (up to 5 cm), but dialysis is still possible; grade 3, completely occluded air filter or dialyzer making dialysis impossible. The coagulation score was also used as a criterion to assess the efficacy.

### 2.5. Calcium Ion Level Analysis

The changes of calcium ions before treatment, 2 h after treatment, and after the completion of treatment, the front of blood pump and intravenous pot, and behind the intravenous pot were observed and recorded in the two groups. And blood calcium level at different time points and in different groups was analyzed using generalized estimating equations.

### 2.6. Safety Evaluation

The adverse reactions were recorded in both groups during dialysis, including perioral numbness, palpitation, convulsion, muscle spasms, and other symptoms.

### 2.7. Statistical Analysis

Statistical analysis was performed using SPSS 22.0 software (SPSS Inc., Chicago, USA). Continuous variables were summarized as mean ± standard deviation (SD) and analyzed with the *t* test between two groups. Qualitative data was described by frequency and corresponding percentages, and differences between groups were compared by a chi-square test. *P* < 0.05 was considered statistically significant.

## 3. Results

### 3.1. General Information of Patients

There were no statistically significant differences between the two groups in terms of gender, vascular access, dialysis age, cause of dialysis for RCA, hematocrit before hemodialysis, hemoglobin, and platelets (Table 1), indicating reliable grouping.

### 3.2. Comparison of Dialysis Adequacy between the Two Groups

At the end of dialysis, spKt/v was analyzed in both groups to determine dialysis adequacy. The results showed that there was no significant difference in spKt/v between patients in the single pump group (1.27 ± 0.13) and patients in the double pump group (1.34 ± 0.26), and the dialysis in both groups was adequate (Figure 2).

### 3.3. Coagulation during Dialysis in Both Groups

The coagulation in the dialyzer and intravenous pot during dialysis was analyzed in both groups. It was found that no severe coagulation occurred in the dialyzers of patients in both groups, and there was no significant difference in the number of mild and moderate coagulation. However, the coagulation in the intravenous pot of patients in the double pump group was significantly lower than that in the single pump group (Table 2).

### 3.4. Comparison of the Safety of Dialysis Treatment between the Two Groups

The safety of anticoagulation during dialysis was evaluated by the level of serum calcium and adverse reactions during dialysis. Blood calcium level at different time points was first analyzed in both groups of patients using generalized estimating equations. The results displayed that RCA reduced blood calcium level at multiple time points, and the double pump group had significantly lower blood calcium level after 2-hour dialysis in intravenous pot than the single-pump group. However, after the completion of dialysis, the serum calcium level basically returned to the pretreatment level (Figure 3). In addition, adverse reactions in all patients after dialysis were observed. It was found that all patients had no obvious perioral numbness, palpitation, muscle twitching, and other discomfort during dialysis.

In the abscissa, 1 represented the front of blood pump and before treatment, 2 represented 2 h treatment and the front of blood pump, 3 represented 2 h treatment and behind filter, 4 represented 2 h treatment and behind intravenous pot, 5 represented before the end of treatment and the front of blood pump, 6 represented after the end of treatment and behind filter, and 7 represented after the end of treatment and behind intravenous pot.

## 4. Discussion

In dialysis patients with high-risk bleeding heparin contraindications, citrate has been shown to be efficacious, and its coagulant effects are mainly in the extracorporeal circulation [7]. However, there is no strict dialysis protocol for RCA, so we observed whether dual pumps could obtain better anticoagulation in hemodialysis. Our study found no difference in coagulation between the single and double pump groups in the dialysis pool. However, in the intravenous bubble pool, the coagulation rate was significantly lower in the double pump group, confirming that double pump operation reduces coagulation in the intravenous bubble pool during dialysis in patients.

It has been suggested that the calcium citrate complex can be rapidly metabolized in the body 30 min after stopping the infusion of citrate [14]. The completion of citrate 0.5-1 h before the end of dialysis is called sequential anticoagulation. In this study, the blood flow was set as 200 ml/min, the ratio of citrate/blood flow was 1.3 in the single pump group, and the ratio of citrate for the front of dialyzer and intravenous pot was 2 : 1 in the double pump group. Then, at the last hour before the end of dialysis, the citrate was discontinued, and after that, the sequential anticoagulation was performed by adjusting the blood flow to 250 ml/min according to the condition of patient. The results showed that there was no severe coagulation in the dialyzers of the two groups, and the coagulation had no significant difference. In the study of Xi Chunsheng on S-RCA [16], the ratio of citrate and blood flow was set as 1.0-2.0. Specifically, on the basis of continuous drip of 4% sodium citrate solution in front of the dialyzer, 10% volume of sodium citrate accounted for the dialyzer front was continuously dripped into the intravenous pot. And the effective rate of anticoagulation in the dialyzer and intravenous pot was 98.7% and 75.5%, respectively, which was similar to our study. In addition, the effective anticoagulant rate of intravenous pot in this study was 98.15% and 100% in single pump and double pump, respectively, which was much higher than 75.5% in the above study.

Several studies [17, 18] have suggested that coagulation in the intravenous pot is the most important reason why RCA does not complete the prescribed dialysis. Therefore, in this study, the effective anticoagulant rate of intravenous pot was high, especially in the double pump group. The difference may be because 1/3 of the citrate volume in this study was infused in front of the intravenous pot, while in the above study, the citrate volume was only 10%. The above result indicated that the ratio of citrate in dual pump may be effective in increasing the anticoagulation rate of the intravenous pot. A prospective study [10] used 4% sodium citrate anticoagulant to pump extracorporeal circulation from the arterial line at 300-375 ml/h (2.0-2.5 times of the blood flow rate). Specifically, a total of 400 hemodialysis treatments were performed, 396 cases completed 4 hours of dialysis anticoagulant therapy, with an overall effective rate of 99%, 4 cases occurred grade III coagulation, and the machine was terminated 3 hours and 30 minutes after dialysis, accounting for 1% (4/400). In the above study, single-pump citrate anticoagulation could also achieve an effective anticoagulation rate of 99%. However, the effective anticoagulation rate of the above study was related to the large amount of citrate application in patients, including 4% citrate at 300-375 ml/h, the blood flow at 150 ml/min, 2.0-2.5 times of the citrate blood flow ratio, and the application of citrate for the whole process. Although the effective anticoagulation rate of the above study was similar to our study, the citrate dosage in the above study was twice that of our study, greatly increasing the ultrafiltration load of patients.

Safety and adequacy of anticoagulation are reflected by monitoring serum calcium ion concentrations for the circulation *in vivo* and *in vitro* in the operation standard of continuous renal replacement therapy. With the long-term progress of dialysis, patients are prone to aortic vascular calcification, and this affects hemodialysis, thereby causing the failure of treatment [19]. Adequate anticoagulation can only be achieved by adjusting the dosage of sodium citrate to maintain the concentration of calcium ions at 0.25-0.35 mmol/L during extracorporeal circulation. Studies have shown that the Ca2^+^ concentration behind the filter reaching 0.25-0.35 mmol/L is not a strict criterion for effective anticoagulation in general dialysis [20]. In this study, it was observed that after dialysis for 2 h, the blood calcium level of patients behind the dialyser in the single pump group was (0.72 ± 0.10) mmol/L, and that of patients in the double pump group was (0.75 ± 0.09) mmol/L, both achieving excellent anticoagulant effect of dialyzer. Another study [21] observed that, if the Ca2^+^ concentration in front of the intravenous pot was over 0.90 mmol/L, most of the dialysis could still be performed successfully. Therefore, the effective blood calcium level behind the filter in general hemodialysis needs further exploration. There are few studies on the effective blood calcium level behind the intravenous pot. In this study, the blood calcium level after 2 hours of intravenous pot dialysis in the double pump group was much lower than that in the single pump group. The result of this study may be because the effective anticoagulant rate of the intravenous pot, and the anticoagulant effect at all levels in the double pump group was better than those in the single pump group. Additionally, after treatment, the serum calcium level of patients was decreased. The decrease of serum calcium level in the double pump group was higher than that in the single pump group, but the serum calcium level of patients *in vivo* in the two groups basically returned to the pretherapy after the end of dialysis.

In this study, sequential anticoagulation was performed with a blood flow setting of 200 ml/min and a citrate/blood flow ratio of 1.3 times, and the kt/v was higher than 1.2 in both groups of patients, showing good anticoagulant effect and safety. And compared with single pump group, the effective rate of coagulation of intravenous pot was significant in double pump group. The optimal dosage of anticoagulation for hemodialysis is to achieve effective anticoagulation with the lowest anticoagulant. A prospective randomized controlled study [22] showed that low-dosage citrate (0.75 times of citrate/blood flow ratio) was not inferior to high-dosage citrate (1.3 times of citrate/blood flow ratio) for anticoagulation effect. Besides, some studies [12, 23] have suggested that in addition to citrate/blood flow ratio affecting the extracorporeal anticoagulant effect of citrate in general hemodialysis, blood flow, ultrafiltration rate, presence of diabetes, and hematocrit are also independent influencing factors for the anticoagulant effect. The reasons why the effective rate of anticoagulation in this study was higher than that in most previous studies were shown as follows: appropriate citrate/blood flow ratio; patients with ultrafiltration volumes higher than 3000 ml were excluded to control the ultrafiltration rate; bleeding patients were included, so baseline hematocrit was not high; and standardized training of the nursing team before research. Based on this study, the analysis for larger scale and some subgroups is needed to further explore the citrate dosage at the next stage of research.

## 5. Conclusion

The double-pump constant citrate sequential anticoagulation mode has a good anticoagulant effect compared with the single-pump therapy. And with the advantages of simplicity, safety, and effectiveness, double-pump therapy in the dialysis process can provide a reference for hemodialysis anticoagulation regimen in end-stage renal disease patients with bleeding in clinical practice.

## Figures and Tables

**Figure 1:** Schematic diagram of single pump and double pump sequential anticoagulation for general hemodialysis treatment using citrate anticoagulation with calcium-containing dialysate.

**Figure 2:** Comparison of spKt/v after dialysis between the two groups.

**Figure 3:** Comparison of blood calcium values at different time points of dialysis between the two groups.

**Table 1:** General information of patients.

	Single pump (*n* = 17)	Double pump (*n* = 15)	*P* value
Gender (male/female)	10/7	7/8	0.492
Age (year)	57.18 ± 13.58	54.47 ± 17.15	0.622
Dialysis age (year)	4.53 ± 2.14	5.6 ± 2.63	0.214
Vascular access			
Internal arteriovenous fistula	15	14	
CUFF catheter	2	1	0.621
Cause of dialysis for RCA			
Trauma	3	2	
Active bleeding	14	13	0.737
Hematocrit (%)	27.29 ± 4.81	28.38 ± 5.22	0.534
Hemoglobin (g/L)	88.80 ± 15.67	92.47 ± 17.16	0.542
Platelets (×10^9^/L)	108.29 ± 13.44	110.80 ± 9.08	0.547

Note: RCA: regional citrate anticoagulation.

**Table 2:** Comparison of coagulation of dialyzer and intravenous pot between the two groups.

	Dialyzer		Intravenous pot	
Score	Single pump	Double pump	Single pump	Double pump
0-1	53 (98%)	47 (94%)	42 (77.78%)	48 (96%)
2	1 (2%)	3 (6%)	11 (20.37%)	2 (4%)
3	0	0	1 (1.85%)	0
*P* value	0.28		0.024∗	

Note: ^∗^*P* < 0.05 vs. single pump group.

## Data Availability

The data used to support the findings of this study are available from the corresponding author upon request.
